The article "Bifrontal Craniectomy: A High-Yield Surgical Training Tool" was published in 2024. Journal: Cureus.

# Bifrontal Craniectomy: A High-Yield Surgical Training Tool

**DOI:** 10.7759/cureus.75533

**Published:** 2024-12-11

**Authors:** Julian M Burwell, Alejandro Bugarini, Mathangi Rajaram-Gilkes

**Affiliations:** 1 Department of Medical Education, Geisinger Commonwealth School of Medicine, Scranton, USA; 2 Department of Neurosurgery, Geisinger Medical Center, Danville, USA

**Keywords:** bifrontal craniectomy, decompressive craniectomy, kjellberg procedure, neurosurgical training, surgical education

## Abstract

Bifrontal decompressive craniectomy (DC), which was once a popular technique for treating midline mass lesions, has seen a notable decline in its therapeutic use within modern neurosurgery. Despite its diminished clinical use, the procedure offers considerable value as an educational tool for surgical training.

This study used a Thiel-embalmed cadaver to demonstrate the bifrontal DC procedure, including a Souttar incision, strategic (MacCarty, zygomatic, and apical) keyhole/burr hole placement, superior sagittal sinus suturing, left frontal lobe decortication, and microscopic visualization of the anterior cranial fossa.

The procedure demonstrated educational value in three ways: first, wide anatomical exposure enables a detailed discussion of tissue handling. Second, an efficient training paradigm that allows multiple surgical techniques to be taught within a limited timeframe. Third, it offers risk management training focusing on superior sagittal sinus protection.

While bifrontal DC has selective therapeutic applications, its potential as a teaching tool is undervalued. The procedure's wide exposure creates an ideal platform for surgical education, allowing residents to develop skills in a structured environment. We advocate its use in training programs by focusing on its educational benefits rather than its limited therapeutic role.

## Introduction

Decompressive craniectomy (DC) has its roots in ancient surgical practices, evolving from Hippocrates' trepanation to contemporary techniques that address intracranial pressure elevations in traumatic brain injury and resection of midline mass lesions [1]. The fundamental principles of trepanation have been adapted into the modern-day Monroe-Kelli doctrine [2,3]. As a fixed space, the brain remains intrinsically vulnerable to pressure changes within the cranium, such as with mass lesions or osmotic changes [4]. From this axiom, the modern-day DC was developed, which entails a calvarial osteotomy to decompress the brain in patients with varieties of intracranial hypertension.

Dr. Raymond Kjellberg first described the bifrontal DC in 1971 [5]. At that time, only 18% of the patients with frontal contusions survived. Owed to the inherent bi-hemispheric decompression of the technique, he argued that the approach was superior to the more popular unilateral decompression. Since then, no further studies have been systematically performed to establish its independent efficiency, and the technique has been largely abandoned, with its use almost exclusively for bifrontal contusions or frontal mass lesions. Here, we reassess the efficacy of bifrontal DC as a comprehensive teaching tool that encompasses surgical skills such as relevant anatomical relationships and risk management scenarios in a single useful procedure.

Educational applications in surgical training

While the therapeutic applications of bifrontal DC have become increasingly focused on specific clinical scenarios [6-8], its potential as a teaching tool remains underexplored in the literature. Neurosurgical program directors frequently face balancing essential clinical responsibilities with dedicated educational time in the new system [9]. Traditional anatomical training often competes with clinical duties, necessitating educational activities yielding high content-to-time ratios to justify time spent outside patient care. While studies have shown that dedicated anatomy lab time is useful for residents and improves evaluation scores, there are limited studies on its efficacy [10,11].

We propose that the procedure detailed below offers educational value through its integrated approach to surgical anatomy. This method allows for the simultaneous instruction of multiple pathologies and surgical techniques, which is impossible to achieve in clinical practice. In this way, the cadaveric laboratory setting provides unique advantages for trainees, enabling deliberate practice and exploration of anatomical relationships without the time constraints and risks inherent to the operating room.

The educational value of bifrontal DC stems from three characteristics. First, the procedure's wide exposure provides direct visualization without the barriers of surgical positional planning [12]. Second, the position offers the possibility of integrating multiple procedures within a single teaching session. Third, the procedure's inherent complications offer an opportunity for risk-management discussion. By performing anatomical dissection, we demonstrate the educational potential of the bifrontal DC by illustrating its application across diverse neurosurgical pathologies.

## Technical report

Our cadaver was selected based on two criteria: (1) it was preserved in a way that is accessible for most academic institutions, and (2) it did not have any prior cranial work despite extensive abdominal and bilateral upper extremity dissection. For surgical education, few criteria are ideal due to the intrinsic nature of variant anatomy in real-life surgical practice. There is no ideal specimen in surgical education.

Specimen preservation

Our lab utilizes mixed preservation techniques: cryopreservation and Thiel embalming. Cryopreservation is employed for specimens the neurosurgery team can use for endoscopic procedure practice. Cryopreservation ensures the most lifelike neuroanatomy and is ideal for preserving the textural quality of connective tissue, such as the calvarial aspects of the meningeal dura, the periosteum, and galea, which can be utilized to support homeostasis and supplant dural loss in bifrontal surgery with a live subject but loses its integrity in Thiel-embalmed subjects [13]. Thiel embalming (ethylene glycol, ammonium nitrate, potassium nitrate, sodium sulfate, boric acid, and trace amounts of formaldehyde), a more cost-effective technique, is used for the gross anatomy lab specimens for the preclinical medical students at our institution [14].

The cadaver used in our study was a Thiel-embalmed cadaver stored at 30ºF from October 2020 (year of death) until July 2023, where it was used for five months of gross anatomy lab dissection prior to the teaching demonstration described.

In our specimen, Thiel embalming techniques preserved the brain parenchyma, neurovascular structures, and cutaneous muscles. While Thiel embalming is effective for preserving neuroanatomy, it presents challenges in maintaining the lifelike characteristics of connective tissue structures such as the meningeal dura, periosteum, and loose connective tissue of the scalp, where the periosteum and dura tended to "flake off" once oxidized. While cryopreservation is a superior method of cadaver storage for dural integrity (such as in dural opening and suturing), given that our approach emphasizes the bony work required in a bifrontal approach, we do not see Thiel embalming as a limitation for institutions hoping to replicate this demonstration due to the cost change and transportation challenges associated with cryopreservation. However, we suggest that Thiel-embalmed subjects remain stored at 30ºF when not in use to preserve the lifelike character of the tissue, and room temperature exposure should be limited to the time of the procedure. If timing is an issue for teaching institutions, the procedure is broken into two sessions: (1) cutaneous dissection, including temporalis fascia removal and careful inspection of vascular structures, and (2) osteotomy with inspection of meningeal dura, superior sagittal sinus, durotomy, and frontal lobectomy. Uncareful dissection and observation may impact clinical practice, and specimen quality is warranted in the context of CT structures. In our experience, elevated cadaveric temperature exposure should be minimized to less than six months at maximum, and less than two months is ideal for Thiel embalmed specimens.

Cadaveric technique

First, a standard bicoronal (i.e., Souttar) incision was made [15]. An incision is carried medial-to-lateral until the superior temporal line is reached. At this point, blunt dissection is performed just at the level of the superficial areolar tissue plane. A Langenbeck elevator is introduced in this plane, and a sharp skin incision is carried down to the level anterior to the tragus. Subsequently, the parietal branch of the superficial temporal artery is identified, coagulated, and divided sharply. Next, the temporalis fascia is incised sharply, and in vivo, muscle fibers are cauterized down to the bone. The deep vascular temporalis fascia is dissected freely off the bone using a Penfield 1 dissector in a superior to inferior fashion along the muscle fibers to reduce subsequent atrophy and wasting. A single myocutaneous flap is elevated antero-inferiorly, paying special attention to the frontalis branch within the fat pad. Either of these effects can cause patients psychological harm following cranial surgery and can be avoided with careful dissection [16].

Once the bones are exposed, burr holes can be made with a high-speed electric cranial drill with an attached cranial perforating bit in the following locations: (1) bilateral burr holes placed at the keyholes as described by MacCarty [17], (2) keyholes drilled bilaterally above the root of the zygomatic arches (Figure 1), and f final burr hole 1 cm posterior to the bregma (Figure 2).

**Figure 1:** Bifrontal approach The bifrontal approach requires the placement of five total burr holes. Two bilateral at the modified keyhole of MacCarty (pink, 1-2 mm posterior to traditional placement), two drilled above the root of the zygoma (posterior to the pterion), and one apical burr hole placed one centimeter posterior to the bregma. Image Credit: Authors; created in BioRender.com

**Figure 2:** Superior oblique view of the specimen Our specimen has a pilot hole drilled in the anterior midline. This is not a part of the procedure.

Unlike previously described approaches, we suggest a single burr hole posterior to the coronal suture. The rationale behind this modification is twofold: in practice, it aims to decrease the reconstruction required by the surgical team and to safeguard the dural sinus from potential damage in the event of an inaccurately positioned burr hole on the superior aspect of the skull. Additionally, a posteriorly placed apical burr hole will preserve a patient's hairline and provide an optimized cosmetic outcome.

It is safest to drill directly above the superior sagittal sinus. In the unfortunate event of a sinus laceration, it is imperative to excise the surrounding bone first to accurately assess the extent of the injury, necessitating quick surgical intervention. If an unfortunate injury to the superior sagittal sinus occurs, it will be the last step, minimizing the time needed for accessibility. Therefore, it is recommended that the maximum amount of bony work be performed first.

The burr holes were connected in the following fashion: (1) first, cut from the apical burr holes to the zygomatic burr holes; (2) second, from the zygomatic burr holes to the keyholes of MacCarty; and (3) finally, connect the keyholes of MacCarty to bisect the frontal bones anteriorly.

Our approach anchors on the keyholes to minimize the possibility of the blade getting pinched while moving along the posterior cutline and to preserve the dura in keeping with the dogma of neurosurgery to cut away from the sinuses. Incisions in the posterior aspect must be made as wide as possible. This method preserved the dural integrity of the specimen without perforation.

Next, the bone must be removed bluntly, which can be challenging due to the dural adherence from the embalming process. Additionally, with the bone piece in a crescent shape, there is more surface area from which the piece must separate. Careful attention must be directed towards this step in the operating room.

The dura did not remain in one piece during the bone removal in our demonstration. Therefore, the dura was used as a teaching tool to indicate suturing of the dural sinus in the case of sinus laceration, as indicated by the suture seen in Figure 3.

**Figure 3:** Superior operative view of the removed bifrontal craniectomy

Next, a left frontal lobectomy with ventricular preservation was performed. Frontal lobe decortication (FLD) is used for intractable frontal epilepsy where patients are resistant to drug therapies [18]. By separating aspects of the frontal lobes, this procedure aims to maximize gray matter resection, avoid damage to motor areas, and preserve the frontal horn of the lateral ventricle. This procedure broadly followed a five-step process as outlined by Wen et al. [19].

A Leica M530 OHX precision surgical microscope (Leica Microsystems, Wetzlar, Germany) was employed in our demonstration, and FLD was performed using the following steps: (1) in vivo coagulation or electrocautery of arterial branches was conducted on the lateral surface of the lobe, which is not a concern in cadaveric studies; (2) a paramedian resection was performed approximately 3 cm caudal to the precentral sulcus, extending to the angle of the corpus callosum; (3) sharp resection began on the gray matter of the lateral surface, with careful attention to avoid the frontal horn of the lateral ventricle; (4) the gray and white matter were removed while preserving the basal surface and olfactory tract; and (5) the entire section was removed, ensuring preservation of the medial surface beneath the rostrum of the corpus callosum. The removed lobe measured approximately 55 × 35 × 22 mm (Figure 4).

**Figure 4:** Close-up views of the resected left frontal lobe

Following careful resection of the frontal lobe, the anterior fossa can be clearly visualized without the need for a surgical microscope. On examination, a saccular bifurcation aneurysm was observed at the M2 segment of the left middle cerebral artery (Figure 5).

**Figure 5:** Magnified superior view of cerebral vasculature and anterior fossa

A recent two-year meta-analysis of global population trends on unruptured intracranial aneurysms (UIA) shows a 5% incidence rate [20]. Of these 5%, significant risk factors contributing to UIA included large vessel occlusion (OR = 1.22, 95% CI = 1.01-1.47) and hypertension (OR = 1.45, 95% CI = 1.24-1.69).

## Discussion

Educational value and applications

Historically, neurosurgery has been limited by the ability to generate meaningful RCTs due to the nature of the conditions treated. In lieu of trials, firsthand experience in an apprenticeship model has long been used to disseminate knowledge throughout the neurosurgical community. This procedure particularly exemplifies the apprenticeship model's strengths by providing wide exposure for anatomical understanding, multiple opportunities for technical skill progression, and structured experience in risk assessment and management. Early exposure to these interventions and discussions with clinicians is highly beneficial for medical trainees at all levels of education. In our institution, these sessions are open to a limited number of medical students, which can assist in integrating their preclinical curriculum into future training. Additionally, residents might find valuable insight into variations in anatomy and learn to be mindful of these in real patients they will encounter. Such knowledge can help to reduce surprises during the surgical procedures they eventually perform.

Anatomical teaching points

Our specimen's aneurysm finding demonstrates the procedure's value in teaching anatomical relationships. Despite being regular in shape, the aneurysm's location distal to the bifurcation point from the left internal carotid artery at the M2 segment presents a unique finding worthy of presentation. This finding provided a teaching opportunity regarding the incidence and etiology of patients with UIAs who face an increased risk of both ischemic and hemorrhagic stroke. A hemorrhagic stroke from a ruptured cerebral aneurysm can be triggered by a refractory period of hypertension, which affects 48% of the US population [21]. Prior to the advent of mechanical thrombectomy, patients with ruptured cerebral aneurysms often met the criteria for emergent craniectomy.

Further reinforcing the anatomical learning objectives, the presence of multiple anatomical variations in this specimen, including bilateral high division of the brachial artery, abnormal course of the ulnar and radial arteries, and bilateral variation in the route of the median nerve [22], created additional teaching value. While observing several such variations in one specimen is uncommon, it highlights the importance of anatomical variation recognition in surgical education.

Future educational applications

While the bifrontal approach may not be optimally suited for pathologies that are laterally positioned when the patient's head is maintained in a static, neutral position, we hypothesize that the bifrontal approach could potentially offer expanded utility in the teaching of midline pathologies in cadaveric specimens.

Future research endeavors could focus on developing structured educational protocols in three key areas: (1) anatomical exposure, with an emphasis on teaching the management of severe aneurysm rupture near the sella turcica; (2) technical skill development, including approaches to skull base mass lesions such as craniopharyngioma; and (3) risk management training, incorporating discussions on falx treatment in central ostomies and technical skills for cutaneous dissection in the temporal regions. Notably, we identified superior sagittal sinus perforation and its management as an underrepresented topic in medical literature. While one case report from 2022 addresses this issue in the context of penetrating head injury, there is a significant lack of literature on iatrogenic causes of superior sagittal sinus laceration [23].

These explorations could provide valuable insights into maximizing the educational benefits of the bifrontal approach in these contexts, further strengthening its role as a wide teaching tool.

## Conclusions

While the bifrontal DC has a narrow therapeutic index, our work demonstrates its unique value as a teaching tool, maximizing exposure and highlighting surgical risk management. By integrating multiple procedures into a single session, we propose that the bifrontal approach could be well suited for structured educational experiences for programs with limited time and/or access to an anatomy lab. With the bifrontal’s access to the anterior cranial fossa, frontal lobes, and cerebral vasculature, we found the bifrontal approach particularly effective for progressive surgical education.

Furthermore, we advocate for a collaborative educational framework that optimizes training in bifrontal craniectomy, recognizing that surgical education benefits from procedures that offer comprehensive teaching opportunities even when their clinical applications may be selective. This approach to surgical education fosters innovation while ultimately improving patient outcomes across the spectrum of neurosurgical practice.

## References

[1] Moon JW, Hyun DK (2017). Decompressive craniectomy in traumatic brain injury: a review article. Korean J Neurotrauma.

[2] Panourias IG, Skiadas PK, Sakas DE, Marketos SG (2005). Hippocrates: a pioneer in the treatment of head injuries. Neurosurgery.

[3] Rossini Z, Nicolosi F, Kolias AG, Hutchinson PJ, De Sanctis P, Servadei F (2019). The history of decompressive craniectomy in traumatic brain injury. Front Neurol.

[4] Mansour A, Lazaridis C, Mangat HS (2023). Chapter 88: intracranial pressure: monitoring and management. Hall, Schmidt and Wood’s principles of critical care, 5th edition.

[5] Kjellberg RN, Prieto A Jr (1971). Bifrontal decompressive craniotomy for massive cerebral edema. J Neurosurg.

[6] Schirmer CM, Ackil AA Jr, Malek AM (2008). Decompressive craniectomy. Neurocrit Care.

[7] Sahuquillo J, Dennis JA (2019). Decompressive craniectomy for the treatment of high intracranial pressure in closed traumatic brain injury. Cochrane Database Syst Rev.

[8] Ramayya AG, Sinha S, Grady MS (2019). Chapter 42: neurosurgery. Schwartz's principles of surgery.

[9] Cohen-Gadol AA, Piepgras DG, Krishnamurthy S, Fessler RD (2005). Resident duty hours reform: results of a national survey of the program directors and residents in neurosurgery training programs. Neurosurgery.

[10] Garcia-Tomas V, Schwengel D, Ouanes JP, Hall S, Hanna MN (2014). Improved residents' knowledge after an advanced regional anesthesia education program. Middle East J Anaesthesiol.

[11] Chino JP, Lee WR, Madden R (2011). Teaching the anatomy of oncology: evaluating the impact of a dedicated oncoanatomy course. Int J Radiat Oncol Biol Phys.

[12] Rozet I, Vavilala MS (2007). Risks and benefits of patient positioning during neurosurgical care. Anesthesiol Clin.

[13] Jang TH, Park SC, Yang JH (2017). Cryopreservation and its clinical applications. Integr Med Res.

[14] Hammer N (2022). Thirty years of Thiel embalming-a systematic review on its utility in medical research. Clin Anat.

[15] Souttar HS (1928). Hunterian lecture on new methods of surgical access to the brain. Br Med J.

[16] Park IH, Kwon H, Kim SW (2016). Cryptogenic temporal hollowing. Arch Craniofac Surg.

[17] Tubbs RS, Loukas M, Shoja MM, Cohen-Gadol AA (2010). Refined and simplified surgical landmarks for the MacCarty keyhole and orbitozygomatic craniotomy. Neurosurgery.

[18] Hirata S, Morino M, Nakae S, Matsumoto T (2020). Surgical technique and outcome of extensive frontal lobectomy for treatment of intracable non-lesional frontal lobe epilepsy. Neurol Med Chir (Tokyo).

[19] Wen HT, Da Róz LM, Rhoton AL Jr, Castro LH, Teixeira MJ (2017). Frontal lobe decortication (frontal lobectomy with ventricular preservation) in epilepsy-part 1: anatomic landmarks and surgical technique. World Neurosurg.

[20] Ortiz AF, Suriano ES, Eltawil Y (2023). Prevalence and risk factors of unruptured intracranial aneurysms in ischemic stroke patients - a global meta-analysis. Surg Neurol Int.

[21] (2017). Hypertension Prevalence Among Adults Aged 18 and Over: United States, 2017-2018. https://www.cdc.gov/nchs/products/databriefs/db364.htm.

[22] Rajaram-Gilkes M, Burwell J, Barr K, Marcincavage D, Fung K, Chukwuemeka E (2023). Bilateral median nerve and brachial artery variations in the arm: a case report. Cureus.

[23] Schlag H, Neuhoff J, Castein J, Hoffmann C, Kandziora F (2022). Rupture of the superior sagittal sinus in penetrating head injury-management of a rare trauma mechanism. J Neurol Surg Rep.

